# Long Distance Metabolic Regulation through Adipose-Derived Circulating Exosomal miRNAs: A Trail for RNA-Based Therapies?

**DOI:** 10.3389/fphys.2017.00545

**Published:** 2017-08-02

**Authors:** Farah Fatima, Muhammad Nawaz

**Affiliations:** ^1^Department of Pathology and Forensic Medicine, Ribeirao Preto Medical School, University of Sao Paulo Sao Paulo, Brazil; ^2^Department of Rheumatology and Inflammation Research, Institute of Medicine, Sahlgrenska Academy, University of Gothenburg Gothenburg, Sweden

**Keywords:** adipose tissue, exosomes, Dicer-knockout, circulating miRNAs, metabolism, lipodystrophy, metabolic diseases, RNA-based therapeutics

## Abstract

The contribution of non-coding RNAs, such as microRNAs (miRNAs) in regulating physiological and pathological states has been intensively elucidated during last 15 years. The discovery of circulating miRNAs (cir-miRNAs) in variety of body fluids, is, however a recent focus of interest in understanding pathophysiological states of their originating cells/organs. Yet another stimulating debate that takes miRNAs to the next level is their presence in exosomes, and this is truly interesting area of research. Exosomes are cell-derived extracellular vesicles, and are naturally equipped biological vehicles that not only enable functional transfer of miRNAs between cells (horizontal transfer) but also foster inter-organ communication, presumably guided by organ specific receptors—decorated on their surface. However, understandings on inter-organ communication elicited by tissue specific exosomal-miRNA fingerprints remain elusive. Recently, Thomou et al., has discovered that adipose tissue contributes a large fraction of adipose specific exosomal-miRNA fingerprints in blood circulation. Experimental evidence emphasize adipose tissue as major depot of cir-miRNAs that sail through blood flow and reach to distal organs—primarily in the liver, where they regulate gene expression of host tissue and elicit metabolic control. This appears to be a genetic form of adipokines (endocrine factors secreted from adipose tissue). We review such offshore metabolic insults, and make an effort to address few important missing links between miRNAs processing and their incorporation into exosomes. We provide potential perspectives on how this knowledge could be steered towards RNA-based therapeutics for monitoring complex metabolic diseases and beyond.

## Introduction

The horizontal gene transfer takes the advantage of transferring genetic material from one cell to other cell (Keeling and Palmer, 2008; Dunning Hotopp, 2011). In higher eukaryotes the mechanism of horizontal gene transfer might have evolved presumably to keep the homeostasis of operational genes (genes participating in housekeeping functions). Jain and colleagues proposed a hypothesis that horizontal transfer of operational genes is a continual process and is far important factor in cellular evolution than previously thought (Jain et al., 1999). However, the horizontal transfer of informational genes (those involved in transcription, translation, and related processes) are far less likely to be horizontally transferred than operational genes (Rivera et al., 1998).

Ratajczak and colleagues were the first to report that microvesicles (nanosized vesicles secreted from cells) may facilitate horizontal transfer of mRNA encoding transcriptional factors that regulate gene expression in recipient cells (Ratajczak et al., 2006). Presumably, this could be considered a transfer of informational genes. Valadi and colleagues for the first time demonstrated that exosomes (40–150 nm nanosized vesicles of endocytic origin) contain microRNAs (miRNAs, miRs) that are transferred between cells horizontally as a mechanism of genetic exchange between cells (Valadi et al., 2007). Albeit, the role of exosomes is well appreciated in mediating genetic communication between cells (Valadi et al., 2007; Mittelbrunn and Sanchez-Madrid, 2012; Nawaz et al., 2016b; Nawaz and Fatima, 2017), however, until recently it remained largely unknown how exosomes could travel between distant organs. In this context, Lyden and colleagues provided captivating evidence that exosomes not only establish intercellular-communication between cells but also foster inter-organ cross-talk guided by organ specific integrins decorated on the surface of exosomes (Hoshino et al., 2015). This and other studies proposed that inter-organ exosomal delivery is tissue specific (Zech et al., 2012; Hoshino et al., 2015). However, identifying miRNA-fingerprints in tissue-specific delivery via exosomes largely remained elusive, until recently recognized in an elegant study by Thomou et al. (2017), that will be the major focus of this review in parallel to few other potential studies which support such mode of gene expression between distant organs.

Fat is a complex, highly variable and heterogenic tissue that appears to have pleiotropic properties and striking plasticity among tissues (Brandao et al., 2017). Adipocyte—a cell that is specialized in storing triglycerides, is the characteristic functional unit of the adipose tissue. Adipose localizes in almost all compartments of the body, constituting subcutaneous inguinal white adipose tissue (WAT), intra-abdominal and epididymal WAT and the brown adipose tissue (BAT) depots (Peirce et al., 2014). In both humans and mice the increased amounts of BAT are associated with a lean phenotype and resistance to development of the metabolic syndrome.

Adipose tissue physiology varies depending on the localization of the fat depot, the cell composition of the tissue and the energy status of the organism which collectively contributing a profound influence on body metabolism (Brandao et al., 2017). Far from being hormonally inert, adipose tissue is recognized as a major endocrine organ and play central role in metabolic regulation through the release of adipokines (cytokines or cell signaling factors secreted by adipose tissue) (Stern et al., 2016). Changes in the metabolic status of the adipocytes affect the production and secretion of adipocyte-derived adipokines. Deregulated metabolism and abnormal distribution of fat in the body leads to major risks of metabolic diseases, such as diabetes mellitus, obesity and lipodystrophy. In obesity the dysregulation of adipose tissue is associated failure in adipose tissue expansion and subsequent storage of surplus lipids and positive energy balance in non-adipose tissues which may result into lipotoxicity a condition which resembles the lypodystrophic syndromes (Slawik and Vidal-Puig, 2007; Virtue and Vidal-Puig, 2010; Mittendorfer, 2011). Lipodystrophy represents fat loss topography, such as general or partial which might be classified as congenital or acquired (Herranz et al., 2008; Chan and Oral, 2010).

The most prevalent form of lipodystrophy is acquired by patients with HIV undergoing antiretroviral treatment (Mallewa et al., 2008; Nolis, 2014). Notably, the highly active antiretroviral treatment downregulates the genes involved in lipid metabolism (Shikuma et al., 2001; Huang-Doran et al., 2010). These patients exhibit higher degree of adipose tissue atrophy and often end up accumulating fat in non-adipose organs, such as liver, skeletal muscles and heart—a phenomenon that is causally linked to the metabolic syndrome (Huang-Doran et al., 2010; Ajluni et al., 2016; Chan et al., 2016). Of particular note, patients with lipodystrophy may represent metabolic impairment by reduction in miRNAs as was recently shown by adipose-derived circulating miRNAs (cir-miRNAs) (Thomou et al., 2017).

## Role of microRNAs in adipose development and metabolic control

MiRNAs are endogenously expressed short non-coding RNAs (ncRNAs) and represent part of the genome that does not code for proteins and play regulatory roles in almost every cellular process through negative control on gene expression (Zeng et al., 2003; Ambros, 2004; Doench and Sharp, 2004; Sevignani et al., 2006; Filipowicz et al., 2008). Several lines of evidence emphasize that developmental events of adipocytes in different fat depots are intrinsically different as a result of genetic regulation. Notably, miRNAs have fundamental role in adipogenesis/differentiation of both brown and beige adipocytes and are central to adipose tissue function and whole body metabolic control in mammals (Mudhasani et al., 2010; Trajkovski and Lodish, 2013; Brandao et al., 2017).

Recent evidence revealed that the expression of components of miRNA processing pathway in adipose tissue (Mori et al., 2012; Oliverio et al., 2016) are highly susceptible to regulation at the level of Dicer. In order to better understand the roles of miRNAs in fat, the mice models lacking Dicer enzyme in adipose issue has been generated using Cre*lox* gene-recombination strategy (Mori et al., 2012). Dicer-knockout mice exhibits a defect in miRNA processing in adipose tissue, resulting in a significant decrease in WAT, the whitening of BAT, insulin resistance and alterations to circulating lipids (Mori et al., 2014). Therefore, changes in adipose-specific miRNAs not only cause impairment of basic functions of adipocytes but also have adipose related deleterious metabolic consequences (Vienberg et al., 2017). However, Dicer-knockout is not the only reason for miRNA dysregulation. In humans, the Dicer levels could be inherently declined due to anomalous body physiology, whereas general down-regulation of miRNAs has been found in human preadipocytes linked to a parallel decrease in Dicer levels with aging (Mori et al., 2012). It emphasizes that the amount of WAT-specific miRNAs decreases with age, owing to a decline in Dicer (Mori et al., 2012). Similar decreases in miRNAs are also observed in humans with HIV-associated lipodystrophy due to decline in Dicer (Mori et al., 2014), against gradual decline in Dicer. In humans, Dicer levels are lower in patients with partial lipodystrophy when compared to healthy individuals, and this is associated with “whitening” and dysfunction of the tissue (Mori et al., 2012; Torriani et al., 2016). Evidence produced from Dicer-knockout *in-vivo* experiments demonstrate that adipose specific Dicer-knockouts exhibit a phenotype that resembles humans with partial lipodystrophy (atrophy of WAT), hypertrophy and “whitening” of BAT, insulin resistance, dyslipidemia, impaired resistance to oxidative stress and premature aging (Mori et al., 2014; Reis et al., 2016).

Recent study provides additional evidence that adipose tissues release miRNAs in the circulation (Thomou et al., 2017). The authors argue that adipose-derived cir-miRNAs are secreted via exosomes at large that travel through blood and regulate gene expression in organs other than adipose. This appears to be novel way of endocrine regulation being far superior to what has been previously thought. However, it needs to determine whether changes in the miRNA processing (owing to Dicer-knockout) will affect the secretion of miRNAs into exosomes. To that end, authors use the mice that are specifically lacking Dicer in adipose tissue and investigate the amount of miRNAs in exosomes and their physiological consequences (Thomou et al., 2017).

## microRNA processing and incorporation into exosomes: missing links

Although the mechanism of miRNA biogenesis and processing has been extensively described, little is known about how processed miRNA are loaded into exosomes. Authors emphasize Dicer-knockout as major strategy to show the altered amount of miRNA secretion into exosomes; however, it is critical to bridge the missing links between miRNAs processing and incorporation into exosomes during the course of exosome biogenesis. Arguably, this missing link will help understand in better way the relevance of miRNAs abundance in exosomes in parallel to action of Dicer (Figure 1).

**Figure 1:** Bridging the missing links between microRNA processing and parallel secretion into exosomes. Schematic representation of different possibilities of miRNA fates in exosomes **(A,B)** in parallel to abnormal procession of miRNAs or Dicer deficit. The blood circulation may acquire both exosomal-fractions and non-exosomal fractions of miRNAs. Those encapsulated in exosomes, travel to long distance organs as protected packages. **(B)** Potential hypothesis of abundance of un-processed pre-miRNAs or empty exosomes against the absence of Dicer enzyme.

Exosomes are synthesized in multivesicular bodies (MVBs) of endosomal compartments which upon fusion with plasma membrane are secreted into extracellular milieu (for detailed mechanisms see Nawaz et al., 2014). We speculate that this process may go side by side to miRNA biogenesis and processing. After being transcribed as long primary transcripts the pri-miRNAs are processed into pre-miRNAs in the nucleus by the enzyme Drosha, a type III endoribonuclease that cleaves the two strands of the hairpin at the stem (Lee et al., 2003; Ha and Kim, 2014), which are then exported to the cytoplasm by exportin proteins (Exportin-5) (Yi et al., 2003; Lund et al., 2004). In the cytoplasm, Dicer enzyme, a type II endoribonuclease cleaves the loop of pre-miRNA and generates miRNA duplex of about 22 base pairs (Lee et al., 2002; Kim et al., 2009). The miRNA duplex is then unwinded and loaded into the ribonucleoprotein complex called RNA-induced silencing complex (RISC) which directs miRNAs to recognize the target mRNA, in order to repress the mRNA translation, or mRNA cleavage and destabilization (Kim et al., 2016).

### Does miRNA processing machinery pave the roads to endosomes?

While it has been shown that major fraction of cir-miRNAs is secreted via exosomes (Thomou et al., 2017), it is rather uncertain what could be the possible mechanism that dictates miRNA selective secretion via exosomes but not the passive leakage from cells? (Figure 1A). Few of the components of RNA-processing machinery were recently proposed for incorporating miRNAs into exosomes. Co-localization and accumulation or re-localization of miRISC components at MVB may favor the processed miRNA sorting into exosomes (Gibbings et al., 2009; Lee et al., 2009; Squadrito et al., 2014). Considering Dicer-knockout, the amount of un-processed miRNAs (i.e., pre-miRNAs) in the cytoplasm must be far higher than processed/mature miRNAs. Therefore, we speculate that exosomes are expected to have higher amount of pre-miRNAs than mature miRNAs (Figure 1B). Since endosomes do not have RISC machinery, therefore the processing of precursor miRNAs within exosomes is ruled out (Chen et al., 2010). However, a recent study argues that exosomes are loaded with RISC-Loading Complex (RLC) and display cell-independent capacity to process pre-miRNAs into mature miRNAs within exosomes (Melo et al., 2014). The incorporation of pre-miRNAs in association with Dicer, transactivation-responsive RNA-binding protein (TRBP) and Argonaute (AGO2) proteins may potentially drive the processing of pre-miRNAs in a cell-independent manner (Melo et al., 2014). If this remains true, then pre-miRNAs might be processed inside exosomes (Figure 1B). However, when Dicer is knocked-out; exosomes will neither have the chance to receive mature-miRNAs from cytoplasm nor the processing of pre-miRNAs inside exosomes as cell-independent manner. Furthermore, we argue that it still remains to be established whether miRNA species in exosomes are abundant in pre-miRNAs or processed mature miRNAs (particularly when cells are knocked-out for Dicer).

## Adipose tissue: a depot of circulating miRNAs?

Although miRNAs have been intensively described in adipose development, little is known about the consequences of cir-miRNA secretion from adipose. In the light of study by Thomou et al. (2017), this section will discuss adipose-derived miRNAs in bloodstream, making an effort to bridge the missing links to exosomes.

### miRNAs in circulation: lipoprotein complexes vs. exosomes

Experimental evidence show that adipose is major source of cir-miRNAs; however it is important also to consider the forms of extracellular-miRNAs (exRNA) other than exosomes. Over the last decade, different forms of secreted exRNA have been reported. This includes both encapsulated in exosomes and non-exosomal forms, such as those secreted in association with RNA-binding proteins and high density lipoprotein complexes (Mateescu et al., 2017). However, pertaining to the presence of exRNA inside exosomes vs. outside exosomes (i.e., non-exosomal exRNA) is a debated issue as there is discrepancy in results shown by different labs (Arroyo et al., 2011; Turchinovich et al., 2011; Gourzones et al., 2013; Chevillet et al., 2014).

In order to present a proof of concept that most of the miRNA is derived from adipose depot, the authors used adipose-specific Dicer-knockout (termed as ADicerKO) and analyzed serum exosomal-miRNA as compared to wild-type mice. In terms of exosomes *per se*, it appears very interesting that the number of exosomes from both ADicerKO-mice and wild-type mice was not much different when examined from per μl of serum. However, to interesting point, what makes the difference between two is the abundance of miRNAs identified in exosomes (reduced in the serum of ADicerKO-mice; Figure 2A). This confirms the initial notion that Dicer-knockout is the major cause of miRNA reduction. The ADicerKO-guided miRNA reduction in circulation is marked as the reduction in exosomal-miRNAs as compared to non-exosomal fractions. Interestingly, it affirms that major proportion of exRNA is chested in exosomes. It is worth mentioning that in Dicer-lacking adipocytes, the loss of exosomal-miRNA secretion is cell-autonomous (i.e., only genotypically mutant cells exhibit the miRNA loss). Keeping in view that Dicer-knockout was adipose tissue specific; therefore, it is safe to affirm that major proportion of cir-miRNA comes from adipose, indicating adipose as major source of miRNAs. What comes physiologically relevant is that several miRNAs that were depleted in ADicerKO serum previously have been revealed to exhibit higher expression in fat (Ortega et al., 2010; Arner et al., 2012; Oger et al., 2014). It further supports the impression of adipose specific origin of cir-miRNAs.

**Figure 2:** Adipose is major source of circulating microRNAs. **(A)** Differences in secreted miRNAs between ADicerKO and wild-type mice. Although numbers of circulating-exosomes are the same in both, however the amount of miRNAs in exosomes from ADicerKO is far less; that is due to Dicer deficit. **(B)** Transplant of brown adipose and serum exosomes from wild-type to ADicerKO-mice reconstitutes miRNA deficit.

### Dicer decline during lipodystrophy: does it mimic dicer-knockout?

As mentioned earlier the humans with impaired metabolism and lipodystrophy exhibit reduction in miRNAs due to disease specific decline in Dicer level (Mori et al., 2014; Torriani et al., 2016). Authors observed that ADicerKO-mice developed a partial lipodystrophy phenotype (a disease characterized by an abnormal distribution of fat by the body). This phenotype is similar to that of humans with congenital generalized lipodystrophy (CGL) and also of patients who developed this condition due to the use of antiretroviral (HIV) treatment. Therefore, it is of particular interest to ask whether the reduced levels of cir-miRNAs are due to impaired metabolism or lipodystrophy in relation to Dicer deficit.

In order to dissociate impaired metabolism from lipodystrophy as major cause of miRNA reduction, it would be important to use mice (control) which have similar metabolic phenotypes to those of ADicerKO-mice. To that end, authors used 4 week old wild-type and ADicerKO-mice, since, at this age, the metabolic phenotypes of ADicerKO-mice are similar to those of wild-type. The serum miRNAs showed reduction in exosomal-miRNAs from ADicerKO-mice as compared to wild-type. It gives the impression that reduction in circulating exosomal-miRNAs is primarily due to miRNA processing rather than the effects of altered metabolism. Consequently, it dissociates altered metabolism from lipodystrophy as major cause of exosomal-miRNAs reduction in circulation.

Correlating such evidence in humans with lipodystrophy or other metabolic diseases would be therapeutically more relevant when considering the application of such tissue specific gene manipulation for therapeutic purposes. In the framework of this attention, it is important to perform exosomal-miRNA profiling on the serum of patients with CGL and compare it with patients having HIV-associated lipodystrophy. The CGL have a generalized loss of adipose tissue; whereas the HIV-associated lipodystrophy patients have decreased levels of Dicer in their fat due to HIV treatment (Mori et al., 2014).

Interestingly, authors show that the amounts of exosomes isolated both from lipodystrophic patients (HIV-patients under treatment and patients with CGL) and controls are the same. But exosomal-miRNAs profiling from lipodystrophic patients showed drastic reduction in amount of exosomal-miRNAs in the bloodstream as compared to controls. This gives the notion that miRNA loss is due to decline in Dicer. It further suggests that it is not the number of secreted exosomes *per se*, that defines the amount of miRNAs, but the processing of miRNA amounts from patient cohorts. From these observations we may infer that the reduction in circulating exosomal-miRNAs primarily reflects the differences in miRNA production (due to declined levels of Dicer) rather than the effects of lipodystrophy itself.

Keeping in view that humans are not Dicer-knockout, but exhibit decline in Dicer due to condition of lipodystrophy; however, Dicer decline mimics the Dicer-knockout in terms of reduction in cir-miRNA levels. Yet, another interesting relevance is that the picture of exosomal-RNA in both patient cohorts is concordant with what was observed in mice having ADicerKO. The serum levels of set of miRNAs that were reduced in mice are also reduced in lipodystrophy patients. Of particular interest, several of these miRNAs have been implicated in the regulation of fat metabolism (Ortega et al., 2010; Keller et al., 2011; Chou et al., 2013).

### Does fat transplantation reimburse the body's dicer deficit?

After having known that ADicerKO-mice exhibit reduction in miRNAs in blood, it would be logically appropriate to ask if fat transplant from wild-type into ADicerKO-mice can reconstitute the levels of secretary miRNAs. In line with this argument, authors transplanted the fat from normal mice into ADicerKO-mice and profiled serum miRNAs of ADicerKO-mice followed by engraftment. Agreeing that if the fat is treasure of miRNAs then WAT and BAT transplants to ADicerKO-mice should in principle, reconstitute the miRNA deficit. As expected, the transplanted fat–mainly BAT significantly restored the circulating exosomal-miRNAs in ADicerKO-mice (Figure 2B). The same was observed when serum exosomes from wild-type were administered to ADicerKO-mice. This supports the idea that adipose tissue is a major source of miRNAs and represents a proof of concept that BAT is the main source of miRNAs.

Notwithstanding, it is paramount to ask whether the pattern of fat distribution has profound influence on metabolism. Revealed from miRNA distribution of transplanted fat depots, BAT depot is shown to play more significant role as compared to inguinal WAT or epididymal WAT. Collectively these experiments reinforce the idea that the distribution of fat depots reflects the adipose physiology. This is particularly true to patients with lipodystrophy, where the pattern of fat accumulation and distribution (atrophy) differs greatly from normal subjects. Interestingly, wild-type BAT transplant into ADicerKO-mice not only reconstituted the Dicer-deficit but also efficiently reversed the phenotypic characteristics, such as glucose intolerance. It could be inferred that BAT is potential source for retaining glucose processing and exhibits pleiotropic effects. Recalling the role of miRNAs in adipogenesis and adipose tissue functions particularly brown and beige adipocytes, the BAT contributes major fraction of miRNAs which regulate fat physiology and metabolism as shown for glucose tolerance and insulin resistance—a potential hallmark of metabolic diseases. From this notion it can be speculated that adipose tissue may also use regulatory messages via exosomes to cope with growing fat mass by inducing glucose tolerance particularly during obesity. However, the glucose tolerance/insulin resistance is not only the result of fat mass expansion and not all forms of obesity result in glucose tolerance. At same body mass index (BMI), both obese and normal-weight individuals may exhibit healthy or unhealthy metabolic profiles (Succurro et al., 2008; Castro et al., 2014). This implies that the morbidly obese individuals (the higher degree of fat mass expansion) are not always insulin resistant; they may also be insulin sensitive. Similarly the lean subjects not always exhibit healthy metabolic profile; they may also represent an unhealthy metabolic phenotype. However, considering the insulin resistance during diabetes the hepatic insulin resistance is a common feature of metabolic diseases, such as type 2 diabetes and lipodystrophy (Moran et al., 2010; Birkenfeld and Shulman, 2014). In such conditions the contribution of exosomes in regulating metabolic profiles and glucose tolerance is a new debate and is truly interesting area of research.

### Long distance inter-organ communication by exosomes: offshore RNA interference?

Arguably, it is interesting to evaluate whether adipose-derived exosomal-miRNAs in the circulation are interfering with the gene expression of other tissues and how such mode of gene expression is followed if miRNA production is impaired by Dicer deficit. In an attempt to provide answer to such argument; first, it is important to understand exosome-mediated gene regulation in other cells (*trans*-regulation between different cell types) by transferring miRNAs from one cell to other (Figure 3; Fatima and Nawaz, 2017). This mode of gene regulation might have evolved in eukaryotes to elicit sophisticated degree of physiological and pathological states.

**Figure 3:** Exosome-mediated *trans*-regulation between different cell types. Exosomes transfer non-coding RNAs between cells and elicit various mechanisms of trans-regulation between cells. Figure originally adopted from Fatima and Nawaz, 2017.

While, periodic observations imply that fat is the major source of cir-miRNAs, nonetheless it would be of great worth to view the physiological and metabolic relevance of miRNAs circulating in the blood. Intriguingly, it will be of utmost importance to argue on those miRNAs that interact with mRNA transcripts of endocrine family of proteins expressed in endocrine organs, such as liver, pancreas, and adipose. To that end, miRNA-mediated regulation of fibroblast growth factor 21 (FGF21) interrogated by Thomou et al. (2017), truly falls under this argument. FGF21 is thought to be expressed primarily in the liver, pancreas and adipose including WAT and BAT (Markan et al., 2014). However, it is also secreted into circulation primarily derived from liver—one of the major center for metabolic affluence. FGF21 is implicated in several metabolic functions, including insulin signaling, glucose uptake, lipid metabolism and food intake (Kharitonenkov et al., 2005). Notably, the secretion of FGF21 in circulation potentially influences metabolism in multiple tissues (Badman et al., 2007; Kralisch and Fasshauer, 2011), whereas deficiency of FGF21 in animal leads to failure of PGC-1α expression and thus exhibit impaired gluconeogenesis and ketogenesis (Potthoff et al., 2009).

Increased *Fgf21* mRNA levels in fat, liver, muscle and pancreas may permit the higher levels of FGF21 secretion into circulation. However, elevated miRNA levels supress the expression of *Fgf21* mRNA and thus FGF21 protein secretion is declined. When miRNA processing is impaired by Dicer-knockout, not only the expression of FGF21 is significantly increased in the liver of ADicerKO-mice but also in the circulating (Thomou et al., 2017). Interestingly, increased FGF21expression in liver corresponds to reduction of exosomal-miRNAs circulating in the serum of ADicerKO-mice. In contrast, the FGF21 expression in the liver of wild-type mice was significantly decreased corresponding to higher levels of exosomal cir-miRNAs. This suggests that adipose tissue sends messages to liver in the form of exosomal cir-miRNAs that regulate gene expression in liver.

To understand this relation, it would be interesting if we correlate circulating exosomal-miRNA levels with liver *Fgf21* mRNA expression and corresponding FGF21 protein secretion in the circulation of ADicerKO-mice after BAT transplant. Following the BAT transplantation, levels of *Fgf21* mRNA in the liver of ADicerKO-mice, as well as the amount of circulating FGF21 were reduced significantly (Figure 4A). Conceivably, one may accept that BAT transplantation has provided some factors(miRNAs) which suppress FGF21 expression that seems to occur at transcriptional level (*Fgf21*-mRNA suppression) regulated by BAT-derived miRNAs. In line with this proposition, the author's hypothesis turns to be true to the edge that circulating exosomal-miRNAs reach to liver and regulate gene expression. The levels of certain miRNAs which are fat-specific, were significantly decreased in the liver of ADicerKO-mice and restored toward normal levels by BAT transplantation. It furthers suggests the idea that BAT-secreted exosomes deliver miRNAs to the liver.

**Figure 4:** Mechanisms of long distance inter-organ cross-talk. **(A)** BAT transplant provides the source of miRNAs in recipient mice that then are circulated to liver where they elicit gene regulation. **(B)** Adipose tissue of ADicerKO-mice is providing no miRNA in circulation, thus allowing the higher expression of FGF2 in liver **(B-i)**, as compared to wild-type which contributes abundance of miRNA in circulation that are delivered to liver and thereby supress *FGf21*-mRNA and thus less secretion of FGF21 protein **(B-ii)**. Transfer of serum exosomal-miRNAs to *in-vitro* settings reflected the corresponding activity of exosomes from ADicerKO-mice (no affect; **B-iii**) and wild-type (reduction of Fgf21 activity; **B-iv**). However, loading of miR-99b into exosomes of ADicerKO-mice mimicked the activity of exosomes from wild-type.

Using bioinformatics tools the potential adipose tissue miRNAs that could target the *Fgf21* mRNA were predicted. Some predicted miRNAs were tested in human liver cells *in-vitro* (miRNA mimic transfection) and evaluated luciferase activity of FGF21. Among these candidates, the miR-99b caused significant reduction in FGF21 who's mRNA (*Fgf21*) was supressed. Notably, these miRNAs are not exosomal-miRNAs–rather are naked miRNAs that were used for transfection. Therefore, this assay does not provide a notion whether this set of miRNAs might also have transferred via exosomes in line with original idea which emphasizes that miRNA transfer to liver is mediated by exosomes. However, this assay at least provides the information that which candidate miRNA is of interest. Thus, exosomes isolated from serum of ADicerKO-mice (lacking adipose miRNAs) can be exogenously loaded with this candidate miRNA and could be co-cultured with liver cells and compare with those from wild-type mice (having adipose miRNAs). By doing so, ADicerKo-exosomes loaded with exogenous miR-99b as well as exosomes from serum of wild-type mice showed reduction in *Fgf21* activity (Figure 4B). This is really interesting to consider that exosomes of ADicerKO-mice loaded with miR-99b significantly inhibited FGF21 similar to exosomes from wild type mice, suggesting that miR-99b is also secreted by adipose tissue into exosomes, and inhibits the expression of FGF21 in the liver. Interestingly, the incubation of liver cells with naked miR-99b does not recapitulate the suppressive effects, whereas those incubated with exosomes, does. This affirms the idea that regulation of FGF21 in liver cells is dependent on exosome based delivery of miRNAs (but this is *in-vitro* transfer).

### Route map from adipose to liver: miRNA troops and exosome vehicles

It is imperative to probe the roads and vehicles to the liver–via blood circulation. The question here is, whether *Fgf21* mRNA is also silenced in liver *in-vivo* and most importantly to ask whether silencing troops (i.e., miRNAs) reached to liver are truly coming from adipose via exosome vehicles. Answers to these questions *in-vivo* would be physiologically more relevant.

Authors performed more elaborative experiments using reporter assays in mice liver to probe if mice have adipose-derived circulating exosomal-miRNAs that target *Fgf21* mRNA. Both ADicerKO-mice and wild-type mice were transfected with FGF21 3′UTR reporter via circulation. Transfected wild-type mice showed reduced FGF21 reported activity since in the circulation it has adipose-derived miRNAs. In contrast, ADicerKO-mice lacks adipose-derived miRNA therefore reporter activity is higher. However, injection of serum-derived exosomes from wild-type mice into ADicerKO-mice suppressed the reporter activity (Figure 5A). Interestingly, following the serum exosome transfer; the recipient ADicerKO FGF21 exhibits same pattern as of donor wild-type. If serum exosomes have miRNAs, such as miR-99b that target *Fgf21-mRNA* and if FGF21′*/*reporter activity is inhibited in the liver, then it indicates that adipose-derived exosomes travel through circulation and regulate FGF21 expression in liver.

**Figure 5:** Adipose-derived exosomes travel through circulation and regulate FGF21 expression in liver. ADicerKO and wild-type mice were transfected with FGF21 3′UTR reporter via circulation **(A-i)**. Wild-type mice show reduced FGF21 reported activity due to presence of adipose-derived circulating miRNAs that is opposite for ADicerKO-mice which lacks adipose-derived miRNA. Upon injecting serum exosomes from wild-type to ADicerKO-mice the recipient ADicerKO-mice mimics the wild-type for reduced reporter activity **(A-ii)**. Since exosomes obtained from serum of ADicerKO lack miRNAs, they are loaded with foreign miRNA-99b and transferred back to ADicerKO which targets *Fgf21*-mRNA and thus reduced expression of FGF21**(A-iii)**; this mimics the activity in in wild-type mice which already has miRNAs **(A-iv)**. **(B)** The expression of human hsa-miR-302f (which does not have mouse homolog) was directly induced in the BAT of mice **(B-i)**, and reporter of hsa-miR in the liver of same mice. BAT-expressed hsa-miR-302f obstructed the activity of reporter in the liver, indicating that adipose (BAT)-specific miRNAs follow the route to liver. **(B-ii)** human hsa-miR-302f expression was induced in the BAT of one mice and reporter in the liver of other mice, and hsa-miR-302f containing exosomes from BAT were injected intravenously to mice having reporter. This results into reduction of reporter activity in the liver of recipient mice. BAT, Brown adipose tissue; ADicerKO, Adipose specific Dicer-Knockout.

Recalling our initial arguments that Dicer-knockout cells may produce empty exosomes? (Recall Figure 1B). If this is true, then empty exosomes obtained from serum of ADicerKO can be loaded with foreign (exogenous-miRNA) and compare with wild-type serum exosomes for their actions on *Fgf21*-mRNA. In separate experiments, authors injected wild-type and ADicerKO-mice with exosomes from ADicerKO-mice, with or without loading of exogenous miR-99b (artificially loaded miRNA in exosomes) (Figure 5A). Administration of ADicerKO-exosomes (so called-empty ones) to ADicerKO-mice did not inhibit reporter activity, meaning that exosomes from Dicer-knockout adipose do not have miRNAs. Interestingly, the administration of ADicerKO-exosomes loaded with miR-99b induced the suppression of the *Fgf21* reporter in ADicerKO-mice accompanied with parallel reduction in hepatic *Fgf21*-mRNA as well as the amount of circulating FGF21.

Arguably, there is an imperative question one may ask whether these miRNAs were already present in the liver (naturally occurring tissue specific miRNAs) of recipient mice that regulate tissue metabolism or they really arrived from other tissue sources. The answer of this uncertainty perhaps remains elusive at least until in line with available literature. This probability could be discriminated by using heterologous miRNA transfer system (i.e., transfer of miRNA from one species to other one, in particular those miRNAs whose homolog is naturally absent in recipient species). To that end, authors used human-specific miRNA (hsa-miR-302f), which does not have mouse homolog. In order to see if adipose-derived miRNAs travel to liver and liver does not already have its own miRNAs of same class; the expression of hsa-miR-302f was directly induced in the BAT of mice to let it be expressed and release into blood stream (Figure 5B). However, the reporter of hsa-miR was not induced in BAT–rather it was induced in liver (but in same mice). If this reporter in liver shows the activity (suppression), it means that hsa-miR expressed from BAT has traveled to liver (as mice liver itself does not have human hsa-miR-302f, means that came from other source that is BAT). As expected, BAT-expressed hsa-miR-302f obstructed the activity of reporter in the liver. This indicates that adipose-specific miRNAs take the route to liver, pointing out the long distance inter-organ communication.

However, it remains to be established whether these miRNA troops are delivered by exosome vehicles? To validate this, authors expressed hsa-miR-302f in the BAT of one mice and reporter in the liver of other mice (Figure 5B). Isolated exosomes from serum of mice expressing hsa-miR-302f from BAT were injected intravenously to other mouse that was transfected with reporter. Interestingly, this exosome-transfer exhibited drastic reduction of reporter activity in the liver of recipient mice, indicating that adipose tissue-derived circulating exosomal-miRNAs regulate the expression in the liver of recipient mice. This is one of the interesting demonstrations from this study that elegantly describes the miRNA interactions between long distance organs and illuminates how exosomes act as abettors and facilitators in this offshore RNA interference eliciting adipose-guided metabolic insults in liver.

## Future perspectives and considerations

Adipose tissue has been known to serve as major endocrine organ and tend to affect the metabolic profiles of other organs by secretory factors, such as adipokines. In principal, fat may have several means to act as endocrine organ, deciphering ectopic and pleiotropic effects conferred in distant organs. However, much sophisticated effects on tissue metabolism shown by cir-miRNAs appear to be newly evolved factors for endocrine functions. Adipose may deploy miRNAs in the circulation (similar to hormones) to serve as genetic form of adipokines for regulating metabolism in distant organs. Exosomes secreted from body organs move through biological fluids and could be harvested as biomarkers (Nawaz et al., 2014, 2016a). Since exosomes are secreted during deregulated metabolism, they could be harvested to predict metabolic profiles of patients with metabolic diseases and may predictive response to therapies. However, applying exosomes and other extracellular vesicles, the sensitive and robust platforms are decidedly required to obtain pure exosomes (Witwer et al., 2013; Nawaz et al., 2014; Mateescu et al., 2017).

Global changes in miRNA biogenesis (as shown by Dicer-knockouts) as well as their concomitant secretion into circulation may reflect the endocrine/pleotropic effects of adipose tissue in the context of systemic regulation of metabolism. Albeit, this study mainly focused on FGF21 regulation in liver; however in a similar way there might be several other potential targets that may help us understand metabolic control in mammals at large.

The phenomenon that the Dicer levels decline with age (aging) and impaired miRNA processing is associated with the development of metabolic diseases (Mori et al., 2012, 2014), may serve as guide to steer current knowledge toward intervening common diseases in the elderly. The current discovery opens new avenues that miRNA deficit could be reversed, perhaps in many organs, to optimize metabolic control. Given that Dicer-knockout mice were shown to develop disorders common in the elderly, such as glucose tolerance and insulin resistance, which were reversed after miRNA reconstitution by BAT. If a patient is deficient for miRNAs and disease pathology is prevailed due to miRNA dependent impaired pathways, this study offers a new way to restore miRNA deficit. Given such importance of miRNAs in adipose tissue, Dicer upregulation may represent a key mechanism to accelerate miRNA production in conditions when these molecules are required at distant locations.

Authors also show, in part, that exosomes can be engineered and loaded with miRNAs of interest and can be delivered to recipient organs. This reinforces the fact that exosomes can be tailored as gene delivery vehicles. Of particular importance, the gene targeting technology, such as Cre/loxP or CRISPR for generating genetically modified mice against human specific diseases, offers an exciting way to refine experimental models in an attempt to bridge the gap between mouse models and human patient studies. The conditional induction or suppression of gene expression of interest in a specific cell or tissue type may help better understand the pathogenesis of disease and determine therapeutic targets. Therefore, the implications of current study, in particular Dicer silencing could be extended beyond metabolic diseases, such as targeting cancers or infectious diseases.

However, exosome tracking in individual diseases would be challenging when intended for the resolution of complex disorders. The heterogeneous nature of particular disease, such as stochastic nature of metabolic diseases and cancers may hinder the consistency to functional readouts of exosomes in therapeutic terms (Fatima and Nawaz, 2015). The additional consideration is the targeting of specific organs, since exosomes have surface chemistries compatible with cell receptors, and thus may interact randomly with off-target cells. Therefore, the uptake and internalization of exosomes by proposed target cells remains an impeding question. Some of the convincing arguments provided by Hoshino et al., are interesting to consider that exosomes could seek target organs through different forms of surface integrins decorated on their surface (Hoshino et al., 2015). However, it would be imperative to find tissue specific miRNA-footprints that may help greatly to intervening organ guided gene therapy. Biodistribution of therapeutic exosomal-RNAs in *in-vivo* models as well as routes of administration needs explicit attention. In addition, defining the doses to each separate disease type and whether the dose-dependent RNA-interference through exosomal-RNAs in model animal experiments is promising must also be determined. If we figure out such options, exosomes might one day be used as safe vectors of RNA-based therapy against multiple diseases.

## Author contributions

FF and MN contributed in conceptualization and writing of the draft, participated in discussions and critical analysis. MN made the schematic illustrations. Both authors agreed and approved the final version for submission.

### Conflict of interest statement

The authors declare that the research was conducted in the absence of any commercial or financial relationships that could be construed as a potential conflict of interest.
